# Application Value of SAT-TB Combined with Acid-Fast Staining in the Diagnosis and Treatment of Pulmonary Tuberculosis

**DOI:** 10.1155/2020/3620425

**Published:** 2020-11-03

**Authors:** Chaochao Qiu, Ning Pan, Yueying Zhou, Hongye Ning, Xinchun Ye, Saiduo Liu, Jichan Shi

**Affiliations:** Department of Infection, Wenzhou Central Hospital, Wenzhou, China

## Abstract

**Objectives:**

This study is aimed at evaluating the clinical application value of RNA simultaneous amplification and testing method for Mycobacterium tuberculosis (SAT-TB) combined with acid-fast staining in the diagnosis and treatment of pulmonary tuberculosis (PTB).

**Methods:**

This paper included 168 suspected and confirmed PTB sufferers admitted to The Sixth People's Hospital of Wenzhou from December 2018 to December 2019, whose sputum was collected and tested using SAT-TB, smear acid-fast staining method, and the BACTEC MGIT 960 system. With the MGIT 960 culture test method as the gold standard, the application value of SAT-TB, acid-fast staining, or SAT-TB combined with acid-fast staining in the diagnosis and treatment of PTB was assessed.

**Results:**

With the MGIT 960 culture as the gold standard, the sensitivity, specificity, positive predictive value, and negative predictive value of SAT-TB for the diagnosis of PTB were 57.3%, 92.5%, 84.3%, and 73.5%, respectively. The conformity was 76.8%, and the Kappa value was 0.515, suggesting a statistically significant difference (*χ*^2^ = 7.314, *p* < 0.05) and a general consistency degree. Additionally, the sensitivity, specificity, positive predictive value, and negative predictive value of SAT-TB combined with sputum smear acid-fast staining were 81.3%, 86.0%, 88.4%, and 80.8%, respectively, with the MGIT 960 culture still the gold standard. The conformity and Kappa value were 83.9% and 0.672, respectively, showing no statistically significant difference (*χ*^2^ = 0.438, *p* > 0.05) and a relatively high consistency degree.

**Conclusion:**

SAT-TB combined with acid-fast staining had a similar detection rate to that of the MGIT 960 culture test with a high consistency degree, which could be applied in the diagnosis of PTB efficiently and accurately.

## 1. Introduction

As a type of chronic infectious disease caused by Mycobacterium tuberculosis (M. tuberculosis), tuberculosis (TB) is able to invade various organs, while pulmonary tuberculosis (PTB) is the most common case [1]. PTB is a major infectious disease severely affecting people's health. There is a large number of PTB sufferers in China, ranking third in the world, only next to India and Indonesia. The principal symptoms of PTB patients are cough, expectoration, fever, fatigue, night sweat, and hemoptysis, and severe symptoms could be fatal [2]. Although its prevalence is gradually falling, PTB remains a significant threat due to its high infectivity [3]. Accordingly, the diagnosis and treatment for PTB are particularly important, and effective PTB control relies on timely diagnosis and treatment. However, the toughest issue at present lies in a lack of early, rapid, and highly specific diagnosis technique during the diagnosis and treatment [1, 2]. Therefore, finding a new breakthrough towards the diagnosis of PTB is an important aspect in PTB control.

Currently, the common diagnosis of PTB is realized by performing a bacteriological examination on sputum and bronchoalveolar lavage fluid (BALF) samples. Mycobacterium culture and sputum smear acid-fast staining are the most common methods, among which the conventional Mycobacterium culture often causes delayed diagnosis and treatment due to the long time required for culture (usually 2 months) [4]. Though the sputum smear acid-fast staining is fast, it is of low sensitivity and is unable to distinguish tuberculosis mycobacterial infection from nontuberculosis mycobacterial infection [5]. It is reported that sputum-negative PTB patients make up 60%-70% [3, 4]. Therefore, the diagnostic ability of these two methods is limited in the clinic.

RNA simultaneous amplification and testing method for Mycobacterium tuberculosis (SAT-TB) combines the technologies of nucleic acid isolation, simultaneous amplification, and testing with fluorescence-labeled hybridization probes. It offers results faster than the conventional bacteriological method, and more importantly, outstanding reproducibility can be achieved with the aid of such technique [6]. Previous research indicated that the specificity of SAT-TB for the diagnosis of PTB is almost 100%, with the sensitivity and accuracy reaching 75.8% and 80.2%, respectively [7], suggesting that SAT-TB as a new detecting method has potential clinical value in PTB diagnosis. Another advantage of SAT-TB is that it targets RNA rather than DNA, and hence, it is capable of detecting live bacteria [8]. This paper was designed to compare the SAT-TB detection technique combined with acid-fast staining with the MGIT 960 culture test and analyze the sensitivity as well as the specificity of SAT-TB or SAT-TB combined with acid-fast staining for PTB diagnosis so as to evaluate their application value in the diagnosis and treatment of PTB.

## 2. Materials and Methods

### 2.1. Research Subjects

This paper included 168 patients (70 confirmed PTB cases and 98 suspected cases) from The Sixth People's Hospital of Wenzhou from December 2018 to December 2019. The cohort was composed of 96 males and 72 females, ranging from 13 to 91 years old, with the average age of 53.8 ± 16.3. Morning sputum samples (*n* = 3) of each patient were collected and tested using SAT-TB, acid-fast staining, and MGIT 960 culture test, respectively. Inclusion criteria for the patients of the study were as follows: [1] diagnosed or suspected PTB sufferers according to the PTB diagnostic criteria, [2] patients with normal liver function, [3] patients with white blood cell count within the normal range, and [4] patients with no history of human immunodeficiency virus infection, acute viral infection, pregnancy, or immunosuppressant medication. Exclusion criteria are the following: [1] patients complicated with other lung diseases, [2] patients with diabetes or hypertension, [3] patients with disorders of consciousness or communication, and [4] patients with poor compliance. This study was approved by the Ethics Committee of The Sixth People's Hospital of Wenzhou.

### 2.2. Reagents and Devices

The M. tuberculosis Nucleic Acid Detection Kit (TB-SAT) (Nos. 20180801, 20181101, 20190301, 20190501, and 20190701), ABI 7500 real-time PCR instrument, and FZP-1 Nucleic Acid Purification Apparatus were ordered from Shanghai Rendu Biotechnology Co., Ltd. The BACTEC MGIT 960 culture system was obtained from Becton, Dickinson and Company (USA). A centrifugal machine was obtained from Hangzhou Xiangrui Technology Co., Ltd. A vortex mixer was purchased from HLD (Taicang, Shanghai, China). A dry bath incubator was ordered from Hangzhou Allsheng Instruments Co., Ltd.

### 2.3. Detection Methods

#### 2.3.1. Sputum Smear Acid-Fast Staining

Sputum smears were placed on a staining rack followed by the addition of basic fuchsin staining solution. After heating to steam and keeping for 5 min, the sputum smears were washed with slow running water; decolorized with destaining solution for 1 min and rinsed; and counterstained with methylene blue for 1 min, washed, and dried naturally. The final smears were positive in red and negative otherwise.

#### 2.3.2. MGIT 960 Culture Test

Five ml of sputum was collected to a 50 ml centrifuge tube with the addition of an equal amount of 2% NALC-NaOH pretreatment liquid. The tube was vortexed for 20 s and left to react for 15 min. With an addition of 50 ml of sterile PBS, the pretreated solution was centrifuged at 3000 g for 15 min, and then, the supernatant was discarded. Thereafter, the solution was added with 2 ml of PBS and mixed. Next, 0.5 ml of the mixture was inoculated in a MGIT culture tube and incubated using the BACTEC MGIT 960 system. If the sample is positive, the red indicating light of the instrument will be on immediately along with an alarm sound.

#### 2.3.3. SAT-TB

Patients' sputum samples were collected every day and sent to Adicon Clinical Laboratories, Ltd. (Hangzhou, China) for SAT-TB detection. The specific procedures were as follows. RNA simultaneous amplification and real-time fluorescence detection were applied. Sputum samples were centrifuged at 13,000 r/min for 2 min with the supernatant discarded, added with 50 *μ*l of sputum liquefying agent, and then oscillated for ultrasonic treatment in an ultrasonic cleaner for 15 min, with the ultrasonic power being 300 W. After ultrasonic treatment was finished, 2 *μ*l of the above fluids was added into a reaction tube containing 30 *μ*l of amplification detection solution, which was then placed in a constant temperature apparatus at 60°C for 10 min followed by 42°C for 5 min. Meanwhile, SAT enzyme solution was also preheated to 42°C. Thereafter, 10 *μ*l of SAT enzyme solution was added to each reaction tube, and the tubes were quickly transferred to a fluorescence quantitative PCR instrument (ABI 7500 FAST) after the solution in tubes was mixed evenly. The constant temperature detecting parameters were set, and the fluorescence detection channel was set as FAM. The PCR reaction was run at 42°C for 1 min, with a total of 40 cycles. The fluorescence signal acquisition channel was set as FAM. The abscissa reading (detection time) of the crossing point of the amplification curve and the threshold curve was dt. dt ≤ 35 meant a positive result, 35 < dt < 40 indicated that a redetection was required, and dt with no reading or equivalent with 40 referred to a negative result.

### 2.4. Statistical Analysis

All statistical analyses were performed using SPSS 19.0 software. With the BACTEC MGIT 960 culture test as the gold standard, we compared the sensitivity, specificity, positive predictive value, and negative predictive value of SAT-TB, acid-fast staining, and SAT-TB combined with acid-fast staining for the diagnosis of PTB. *χ*^2^ examination was adopted, and *p* < 0.05 was considered statistically significant. The Kappa index was used to assess the consistency of the results. The consistency degree was divided into 3 grades according to the Kappa value which, respectively, are low (<0.4), general (0.4-0.6), and high (>0.6).

## 3. Results

### 3.1. Comparison between SAT-TB and Acid-Fast Staining

Among the 168 patients' specimens, there were 51 positive cases (including 8 cases of nontuberculous mycobacterium (NTM)) and 117 negative cases using acid-fast staining. There were 55 positive cases and 113 negative cases tested by SAT-TB. Among the 51 positive cases tested by acid-fast staining, there were 40 positive cases and 11 negative cases detected by SAT-TB. Among the 117 negative cases tested by acid-fast staining, there were 15 positive cases and 102 negative cases detected by SAT-TB. With acid-fast staining being the standard, the sensitivity and specificity of SAT-TB were 78.4% (40/51) and 87.2% (102/117), respectively. The consistency degree of SAT-TB and acid-fast staining was 84.5% (142/168), which demonstrated no marked statistical difference (*χ*^2^ = 0.221, *p* > 0.05). The details are listed in Table 1.

### 3.2. Comparison between SAT-TB/Acid-Fast Staining and MGIT 960 Culture Test

There were 75 positive cases (11 cases had NTM, including 7 Mycobacterium intracellulare, 2 Mycobacterium avium complex, 1 Mycobacterium abscessus, and 1 Mycobacterium kansasii) and 93 negative cases using the MGIT 960 culture test. Among the 75 positive cases tested by MGIT 960, there were 45 positive cases and 31 negative cases detected by acid-fast staining and 43 positive cases and 31 negative cases detected by SAT-TB. Among the 93 negative cases tested by MGIT 960, there were 10 positive cases and 82 negative cases detected by acid-fast staining and 8 positive cases and 86 negative cases detected by SAT-TB. With MGIT 960 being the standard, the sensitivity, specificity, positive predictive value, and negative predictive value of acid-fast staining were 60.0% (45/75), 88.2% (82/93), 81.8% (45/55), and 72.6% (82/113), respectively. The conformity of acid-fast staining and MGIT 960 was 75.6% (127/168), which revealed a significant statistical difference (*χ*^2^ = 5.019, *p* < 0.05). The Kappa value was 0.493, unveiling a general consistency of the results detected by acid-fast staining and MGIT 960. The sensitivity, specificity, positive predictive value, and negative predictive value of SAT-TB were 57.3% (43/75), 92.5% (86/93), 84.3% (43/51), and 73.5% (86/117), respectively. The conformity of SAT-TB and MGIT 960 was 76.8% (129/168), which uncovered a marked statistical difference (*χ*^2^ = 7.314, *p* < 0.05). The Kappa value was 0.515, showing a regular consistency of the results detected by SAT-TB and MGIT 960. The details are listed in Table 2.

### 3.3. Comparison between SAT-TB Combined with Acid-Fast Staining and MGIT 960 Culture Test

Among the 75 positive cases tested by MGIT 960, there were 61 positive cases tested by SAT-TB and/or acid-fast staining and 19 negative cases detected by both SAT-TB and acid-fast staining. Among the 93 negative cases tested by MGIT 960, there were 8 positive cases tested by SAT-TB and/or acid-fast staining and 80 negative cases detected by both SAT-TB and acid-fast staining. With MGIT 960 being the standard, the sensitivity, specificity, positive predictive value, and negative predictive value of SAT-TB combined with acid-fast staining were 81.3% (61/75), 86.0% (80/93), 88.4% (61/69), and 80.8% (80/99), respectively. The conformity of SAT-TB combined with acid-fast staining and MGIT 960 was 83.9% (141/168), which showed no marked statistical difference (*χ*^2^ = 0.438, *p* > 0.05). The Kappa value was 0.672, demonstrating a high consistency degree of the results detected by SAT-TB combined with acid-fast staining and MGIT 960 culture test. The details are listed in Table 3.

## 4. Conclusion

A rapid and accurate diagnosis of PTB is the key for PTB control. Although a Mycobacterial culture test remains the gold standard for PTB diagnosis, M. tuberculosis grows slowly and it requires a long time to produce detection results [9]. Compared with the culture test method, the application of a molecular diagnostic technique in PTB diagnosis is able to quickly detect M. tuberculosis from patients' specimens [5]. With the application and prevalence of molecular diagnostic techniques in recent years, the detection rate of PTB has markedly risen. At present, there are mainly two probe-based molecular diagnostic approaches to PTB. One uses DNA as a template, with the target DNA amplified by PCR to detect DNA products of M. tuberculosis in specimens [6, 7]. Though the application of TB DNA detection considerably raises the detection rate of PTB, DNA as an amplified product can easily spark laboratory cross-contamination and cause false-positive results, thereby leading to errors of clinical diagnosis. Another one uses RNA as a template, with the target RNA amplified by PCR to detect RNA products of M. tuberculosis in specimens [8]. During this approach, RNA is the initial target, and gene contamination can be effectively avoided owing to the fact that RNA is extremely easily degradable, which supports that RNA only exists in live bacteria. As a result, RNA simultaneous amplification and testing are capable of not only serving as an indicator for TB diagnosis but also assessing disease activity and evaluating the effect of treatment.

In this study, morning sputum samples of 168 patients were examined using SAT-TB, acid-fast staining, and MGIT 960 culture system, respectively. With MGIT 960 being the standard, the sensitivity, specificity, positive predictive value, and negative predictive value of acid-fast staining for the diagnosis of PTB were 60.0%, 88.2%, 81.8%, and 72.6%, respectively, which showed a marked statistical difference between the two methods (*χ*^2^ = 5.019, *p* < 0.05), suggesting that the detection rate of PTB by acid-fast staining was lower than that by MGIT 960. Besides, with MGIT 960 being the standard as well, the sensitivity, specificity, positive predictive value, and negative predictive value of SAT-TB were 57.3%, 92.5%, 84.3%, and 73.5%, respectively. The difference was statistically significant (*χ*^2^ = 7.314, *p* < 0.05), revealing that the detection rate of PTB by SAT-TB was lower than that by MGIT 960. A study indicated that for PTB diagnosis, the sensitivity and specificity of SAT-TB were 92% and 86%, respectively, with the detection rate of 54% [10]. In 2012, Cui et al. [10] made a comparison between SAT-TB and MGIT 960 culture test which were used for identification of M. tuberculosis, suggesting that their conformity reached 95.6% and their detection results were similar. The present study demonstrated that the detection rate of PTB by SAT-TB was slightly lower than that by the MGIT 960 culture test. This research collected sputum specimens not only from suspected cases of PTB but also from some confirmed cases who were taking anti-TB drugs. However, SAT-TB could only detect active M. tuberculosis and show no response to dead ones; hence, the positive detection rate was low. Besides, the sputum samples of NTM-infected patients were tested positive using either acid-fast staining or MGIT 960. A part of the research subjects were ultimately identified to be infected with NTM, and their SAT-TB results all presented negative, which contributed to the lower positive detection rate. However, by comparing SAT-TB combined with acid-fast staining with the MGIT 960 culture test, we found that the sensitivity, specificity, positive predictive value, and negative predictive value of SAT-TB combined with acid-fast staining were 81.3%, 86.0%, 88.4%, and 80.8%, respectively, showing no marked statistical difference between the two approaches (*χ*^2^ = 0.438, *p* > 0.05), which revealed that the results of SAT-TB combined with acid-fast staining were similar to those of MGIT 960. The Kappa value was 0.672, demonstrating high consistency of the results between SAT-TB combined with acid-fast staining and MGIT 960. Consequently, it could be concluded that the detection rate of PTB by acid-fast staining or SAT-TB was lower than that by the MGIT 960 culture test, whereas that by SAT-TB combined with acid-fast staining was similar to that by MGIT 960 with a high consistency degree. As a consequence, SAT-TB combined with acid-fast staining is able to not only diagnose PTB efficiently, accurately, and faster as well as cover the shortage of the MGIT 960 culture test that takes a long time to culture but also clarify disease activity and better assess the effect of treatment. For the diagnosis of suspected cases or the follow-up examination of PTB patients after treatment, SAT-TB combined with acid-fast staining can effectively increase the detection rate of M. tuberculosis and help medical staff know more about the disease conditions of patients so as to reduce misdiagnosis and missed diagnosis.

In conclusion, SAT-TB combined with acid-fast staining is able to diagnose PTB efficiently and accurately; hence, it is worthy of clinical promotion.

## Figures and Tables

**Table 1:** Comparison between SAT-TB and acid-fast staining.

SAT-TB	Acid-fast staining		Total
	+	-	
+	40	11	51
-	15	102	117
Total	55	113	168

**Table 2:** Comparison between SAT-TB/acid-fast staining and MGIT 960 culture test.

MGIT 960	Acid-fast staining		SAT-TB		Total
	+	-	+	-	
+	45	31	43	31	75
-	10	82	8	86	93
Total	55	113	51	117	168

**Table 3:** Comparison between SAT-TB combined with acid-fast staining and MGIT 960 culture test.

MGIT 960	SAT-TB combined with acid-fast staining		Total
	+	-	
+	61	19	75
-	8	80	93
Total	69	99	168

## Data Availability

The data and materials in the current study are available from the corresponding author on reasonable request.
